# Computed Tomography Image Segmentation of the Proximal Colon by U-Net for the Clinical Study of Somatostatin Combined with Intestinal Obstruction Catheter

**DOI:** 10.1155/2022/6868483

**Published:** 2022-01-18

**Authors:** Chunpeng Dou, Kuiwu Li, Liang Wang

**Affiliations:** The First Department of General Surgery, Fuxin Centre Hospital, Fuxin 123000, China

## Abstract

**Objective:**

U-Net technology is implemented for image segmentation to diagnose cases of intestinal obstruction. To evaluate the application value of somatostatin combined with transanal intestinal obstruction decompression catheter in the treatment of distal colonic malignant intestinal obstruction and to explore the therapeutic effect of somatostatin on acute abdomen surgery in patients with intestinal obstruction.

**Methods:**

After the segmentation technique, a retrospective analysis of 30 patients with acute and complete distal colonic malignant obstruction treated by surgery was divided into a control group and an observation group according to a random number table. The treatment efficiency, clinical symptoms, disappearance time after treatment, and the incidence of complications were compared between the two groups of patients.

**Results:**

The image segmentation using U-Net can effectively assist in the medical diagnosis of the colon. Our study found that patients with combined treatment with somatostatin and anal intestinal obstruction catheter were relieved of preoperative abdominal pain and abdominal distension; compared with the abdominal circumference at the time of admission, the abdominal circumference was significantly reduced. Abdominal examination was performed 3 days after comprehensive treatment, and combined with computed tomography (CT), we observed that the measured maximum transverse diameter of the proximal colon was significantly smaller than that before treatment. Before treatment, all patients were divided into a control group and a treatment group. After treatment, the symptoms of the two groups of patients were alleviated. The treatment effective rate of the observation group was 93.3%, and the treatment effective rate of the control group was 73.3%. The effective rate was significantly higher than that of the control group, and the difference was statistically significant.

**Conclusions:**

Through the use of image segmentation technology, somatostatin treatment of early inflammatory bowel obstruction after acute abdomen surgery can effectively improve the treatment efficiency of patients, shorten the disappearance of clinical symptoms, reduce the incidence of complications, and have a significant therapeutic effect, which is worthy of clinical application. Somatostatin combined with enteral obstruction catheter treatment is safe and effective for elderly patients with acute distal large bowel malignant intestinal obstruction. It has a higher completion rate of laparoscopic surgery and a first-stage anastomosis power, which reduces the risk of perioperative period and reduces the patient's financial burden.

## 1. Introduction

Many computer vision tasks require intelligent segmentation of images to understand the content of the image and make it easier to analyze each part. Today's image segmentation technology uses deep learning models to accurately understand the real world, which was unimaginable ten years ago. Image segmentation uses a computer to distinguish the content of an image, which is a very challenging task in a computer vision system. Semantic segmentation is to classify all pixels in an image, and pixels with the same semantics are segmented. In recent years, there has been an increasing demand for image segmentation in industries such as smart medical care, autonomous driving, indoor navigation, human-computer interaction, virtual or augmented reality, robotics, image beautification, and smart agriculture. More and more products need to be based on depth. The learned image segmentation algorithm serves as technical support.

In the field of smart medicine, medical image analysis has become a hot research topic. Brain tumor is an abnormal tissue caused by uncontrollable factors that cause cell canceration and proliferation. It seriously threatens human life and health. It is one of the main research contents of the medical scientific research team. Segmentation diagnosis of brain tumors in brain MRI images to determine the exact location of areas such as edema, enhancement, and necrosis plays a key role in later diagnosis and treatment, causing systemic inflammatory response syndrome, sepsis, and even organ dysfunction, making the condition more complicated [1–3]. The traditional brain tumor segmentation method is based on the knowledge of anatomy and pathology by radiologists, with the help of specific software to perform manual segmentation and label the data. This method is time-consuming and labor-intensive, the correct rate of annotation varies due to personal ability, and there is instability. Therefore, traditional brain tumor segmentation methods are difficult to meet the needs of clinical use in terms of segmentation speed and segmentation accuracy. It is particularly important to realize fast and accurate brain image segmentation with the help of a computer.

Intestinal obstruction is susceptible to gastrointestinal flora imbalance. Inadequate treatment or drug-resistant flora can be complicated by bacterial and endotoxin translocations, causing intestinal infections and systemic inflammatory response syndrome and sepsis, and even more, insufficiency of organs makes the condition more complicated [1–3]. How to correct the imbalance of intestinal flora as soon as possible, so that patients can recover quickly, is an important research question. In the past, clinically often highly targeted antibiotics were used to kill or inhibit intestinal pathogenic bacteria. It is expected that probiotic bacteria in the intestinal tract can grow rapidly, but the result is often counterproductive, resulting in the emergence of drug-resistant pathogenic bacteria or serious double infections. Microecological preparations, also known as microecological regulators, are produced with the development of intestinal nutritional support [4–6]. The human intestine is a huge and complex microecosystem, and the balance between its various floras is of great significance to the health and recovery of the disease. Studies have shown that the probiotics inherent in the live intestinal tract can be applied, supplemented with prebiotic preparations (which can inhibit the growth of pathogenic bacteria and promote the growth of probiotics), to achieve the restoration of intestinal flora balance.

Somatostatin is a clinically widely used neurohormone. It is mainly used for hemorrhage caused by liver cirrhosis and has a certain effect on upper gastrointestinal bleeding. Its main role is to inhibit the secretion of growth hormone, glucagon, insulin, and other hormones. In addition, it also affects the absorption of the gastrointestinal tract and nutritional functions. After intravenous injection of somatostatin, it can be quickly metabolized in the liver of the patient, 70% excretion can be achieved within hours, and the effect is fast. The application of intestinal obstruction symptoms is mainly to inhibit the secretion and stasis of gastrointestinal fluids of patients and relieve abdominal distension and abdominal pain symptoms. Relevant research shows that the number of patients with intestinal obstruction treated with somatostatin within 48 hours of emergency treatment is significantly lower than that if patients who are not treated with somatostatin which can effectively improve the intestinal surgical conditions of patients [7, 8]. Somatostatin treatment can effectively reduce the accumulation of digestive juice in the intestine by more than 50%. It can not only reduce the edema of the intestinal lining and maintain the integrity of the intestinal mucosa but also promote the blood circulation of the patient, thereby shortening the treatment time and facilitating the recovery of the patients' health [9, 10].

Computed tomography (CT) examination is fast and has high resolution. With the development of CT technology, thin-layer volume scanning and various image postprocessing techniques have significantly improved the diagnostic performance of CT and are widely used in the diagnosis of intestinal obstruction diseases. Therefore, in this study, CT images can help to analyze the condition of patients with intestinal obstruction.

The traditional conservative treatment methods for intestinal obstruction are fasting, gastrointestinal decompression, and parenteral nutrition support. Among them, gastrointestinal decompression is often performed through the nasogastric tube. Traditional nasogastric tube decompression can only drain the liquid in the stomach cavity, but the fluid in the intestinal cavity cannot be fully drained, causing a large amount of gas and liquid to accumulate in the intestine, causing the intestinal wall to expand and edema, and then blood flow is blocked, affecting the intestine road function recovery. An intestinal obstruction decompression tube is used to insert the catheter through the nasal cavity and esophagus with the aid of gastroscope or X-ray and then suck the stomach contents into the small intestine. The intestinal obstruction decompression tube can more easily pass through the pylorus and enter the intestinal cavity. Intestinal decompression relieves intestinal edema and restores blood flow when decompression is sufficient, laying a good foundation for restoring intestinal function [11].

Therefore, we envisage that if the microecological preparation and the intestinal obstruction decompression tube are jointly applied, the microecological preparation will be injected into the intestinal cavity near the obstruction through the decompression tube after the intestinal tube is fully decompressed, which can effectively inhibit the growth of pathogenic bacteria and prevent it in time. Or correct the intestinal flora imbalance, reduce the application rate of antibiotics, and timely monitor the changes of intestinal flora and endotoxin levels through the drainage fluid, and provide experimental basis for clinicians to choose the timing of surgery. It can also effectively improve the symptoms and signs of patients with intestinal obstruction, improve the cure rate of patients, and shorten the length of hospital stay and has important clinical significance for the prognosis of patients with intestinal obstruction [12, 13]. Intestinal obstruction is a common acute abdomen in gastrointestinal surgery.

With the increasing incidence of colorectal cancer, there are more and more patients with acute mechanical intestinal obstruction caused by colorectal cancer. Most patients also have complications such as dehydration, electrolyte disturbance, and hypoproteinemia, which increase the risk of emergency surgery. Traditional surgical treatment methods include palliative tumor resection and proximal colostomy or only colostomy, which requires a second surgery to close the stoma or second-stage tumor resection, which increases the patient's hospital stay and hospitalization costs. Recent studies have shown that somatostatin can delay the progression of malignant intestinal obstruction and effectively improve the clinical symptoms of patients [14, 15]. The safety and effectiveness of transanal intestinal obstruction catheter for the treatment of colorectal malignant intestinal obstruction have been confirmed [16, 17].

## 2. Materials and Methods

### 2.1. Image Segmentation Based on Full Convolutional Network

A fully convolutional network (FCN) replaces the fully connected layer in the convolutional network structure with a fully convolutional layer, predicts the category of pixels from the extracted feature map, and realizes pixel-level classification or segmentation. The full convolutional network can input images of any scale, which solves the problem of repeated calculation of adjacent pixels. But the shortcoming of the full convolutional network is that the training result is still insufficiently accurate, and secondly, the spatial law is ignored.

U-Net uses the symmetrical connection structure of the codec, which performs well in the field of medical image segmentation. The model structure is shown in Figures 1–3. There are many variant structures of U-Net, such as the combination with modules such as ResNet. V-net has made improvements on the basis of U-Net, using 3D convolution; improving the objective function to the Dice coefficient; using random nonlinear transformation and histogram matching as new data enhancement methods; and adding the residual module increases convergence. DenseNet is applied to a fully convolutional network as a segmentation network. This structure can achieve optimal results without pretraining and postprocessing of conditional random fields, as shown by Figure 4.

SegNeW performs low-dimensional encoding on the input image and then uses the direction invariance of the decoder to restore the image. This will generate segmented images on the decoder side. SegNet and FCN are similar in structure but different in sample mode. FCN uses deconvolution upsampling, while SegNet records the coordinate position of the maximum value during the pooling process. During the upsampling process, the value of the feature map is mapped to the corresponding position, and the feature values of other positions of the new feature map are set to zero. During the sampling process of DeconvNet, both the encoder part and the SegNet adopt the structure of VGG16. The difference between DeconvNet and SegNet is that the network finally adds two fully connected layers.

The above four network structures are similar, and they are both the structure of the encoder and the decoder. The encoder part is a combination of the convolutional layer and the pooling layer. The decoder is an upsampling process. Different network structures mainly differ in upsampling methods. The sampling method of FCN is to add to the feature map after deconvolution. U-Net is the same as the sampling method of FCN. DeconvNet maps the feature value to the new feature according to the position of maximum pooling in the sampling process. In the figure, SegNet is the same as DeconvNet.

One of the main purposes of Deeplab is to perform image segmentation while helping control signal extraction, thereby reducing the number of samples and the amount of data that the network must process. Another purpose is to support multiscale contextual feature learning-to-gather features from images of different scales. Deeplab uses ImageNet pretrained residual neural network for feature extraction. Deeplab uses hole convolution instead of ordinary convolution. The different expansion rate of each convolution enables the residual neural network to capture multiscale contextual information. Deeplab is composed of three parts: hole convolution, which can expand or contract the convolution filter; residual neural network; and Microsoft's deep convolution network, which can pass parameters in thousands of layers of neural networks without losing the parameter characteristics. The powerful representation ability of residual neural network promotes the application of computer vision, such as target detection and face recognition; passive spatial pyramid, used to provide multiscale information, uses a set of convolutions with different expansion rates to capture long-term context. The passive spatial pyramid also uses global average pooling (GAP) to incorporate image-level features and add global contextual information.

### 2.2. Patient Information

Thirty patients with colorectal cancer with incomplete intestinal obstruction who underwent surgical treatment in colorectal and anal surgery in our hospital from September 2010 to November 2016 were selected. The following are the inclusion criteria: (1) preoperative clinical manifestations such as abdominal distension, abdominal pain, and intestinal obstruction. Standing abdominal plain films show intestinal dilation and gas-liquid plane. Colonoscopy or abdominal CT diagnosis of colorectal cancer meets the diagnostic criteria for obstructive colorectal cancer, and patients with colorectal cancer were confirmed by postoperative pathology. According to the random number table method, it was divided into an observation group and a control group. The observation group was given Nengquansu combined with PEG for perioperative intestinal preparation, and the control group was given traditional liquid diet and senna leaves for intestinal preparation (observation group: 15 cases, 8 males and 7 females; age 54~77 years old; obstruction site: 4 cases of rectal obstruction, 6 cases of sigmoid colon obstruction, 3 cases of descending colon obstruction, two cases of colonic splenic flexion obstruction, and 15 cases in the control group, 6 males and 9 females; age 56 to 75 years old; obstruction sites: 5 cases of rectal obstruction, 6 cases of sigmoid colon obstruction, 3 cases of descending colon obstruction, and one case of obstruction of splenic flexure of the colon). Patients with severe heart, liver, and kidney diseases and malignant tumors were excluded. The difference in baseline indicators between the two groups was not statistically significant (*P* > 0.05) and was comparable.

### 2.3. Research Methods

In the intestinal preparation method, the observation group started oral administration of Nengquansu 1 can/d in the first week before surgery, 2/3 in the morning and 1/3 in the afternoon; meanwhile, 1 bag/d of PEG was taken orally every afternoon from the beginning of the week before the operation, two bags were taken orally 1 d before surgery. The control group was given a conventional liquid diet, and at the same time, senna extracts were given (1 g) before surgery (10 g/d); fasting 1 d before surgery, 20 g of senna extracts was given. All patients were not with enema. In the preoperative nutrition scoring method, the European Nutrition Risk Screening Table NRS-2002〔4〕 was used as a nutrition scoring tool to evaluate the preoperative nutritional status of the two groups. NRS-2002 includes two parts: preliminary screening and final screening, and is finally divided into 4 grades: none, mild, moderate, and severe according to the patient's disease severity and nutritional status, which are counted as 0, 1, 2, and 3 points, respectively. Note that ≥3 points indicate that they are at risk of malnutrition and need nutritional support.

The control group was treated with conservative treatment methods, such as fasting before surgery, decompressing the gastrointestinal tract of the patient, correcting the patient's acid-base balance disorder and water and electrolyte disorder, and intravenously injecting dexamethasone and anti-infection according to the patient's specific situation. Treatment, such as taking cephalosporin antibiotics, was used. The observation group was treated with intravenous somatostatin for 3 to 12 days of continuous treatment. The dose was 6 mg each time. When somatostatin was infused, it was injected into 50 ml of 0.9% saline or 5% glucose injection before infusion. Care should be taken to control the rate of infusion to keep it at 2 ml per hour and continue treatment for 3 to 12 days.

### 2.4. Research Indicators

#### 2.4.1. Postoperative Clinical-Related Indicators

The operation time, hospitalization time, tolerance of solid food postoperatively, postoperative anal exhaust time, and postoperative complications were observed in the two groups.

#### 2.4.2. Immunological Test Index

The levels of T-lymphocyte subsets (CD3+, CD4+, CD8+, and CD4+/CD8+) and immunoglobulin (Ig G, Ig M) of patients were detected 1 day before operation and 7 days after operation. The content of serum Ig G was measured by radioimmunoassay, and the content of serum Ig M was measured by enzyme-linked immunoassay. The operation process is strictly in accordance with the instructions of the kit. The percentages of CD3+, CD4+, and CD8+ were measured by flow cytometry (US BD). We took 2 ml of peripheral venous blood in an anticoagulation tube, added 50 *μ*l of anticoagulated whole blood and 20 *μ*l of fluorescent antibody, mixed and placed at room temperature for 30 min, and added 450 *μ*l of hemolysin, mixed and placed at room temperature for 15 min. We then used the automatic analysis software to set the test acquisition conditions. After the quality control is passed, the sample analysis is performed, and the detection percentages of CD3+, CD4+, CD8+, and CD4+/CD8+ are reported.

#### 2.4.3. Observation Index

The effectiveness of treatment, the time of disappearance of clinical symptoms, and the incidence of complications after treatment were compared between the two groups. The evaluation criteria for the effectiveness of treatment are as follows [18–20]:

1. Cure: the clinical symptoms such as abdominal swelling, abdominal pain, nausea, and retching disappeared. The abdominal X-ray examination revealed that the intestinal effusion and gas disappeared, which was regarded as cured.
2. Effective: clinical symptoms such as abdominal swelling, abdominal pain, and nausea and retching have been greatly relieved. The abdominal X-ray examination found that the symptoms of intestinal obstruction have been relieved and are considered effective.
3. Invalid: in the patient's clinical symptoms, there was no relief or even signs of aggravation. The abdominal X-ray examination showed no improvement in the symptoms of intestinal obstruction, which was regarded as ineffective. Total effective rate = (cured + effective) cases/total cases × 100%.

Clinical symptom relief includes abdominal pain relief, time for defecation and defecation, and gastrointestinal decompression. Complications include abdominal infection and peritoneal effusion.

### 2.5. Statistical Processing

SPSS17.0 was used for data analysis, and the count data was expressed in the form of mean ± standard deviation (mean ± SD). The comparison between the two groups used Student's *t*-test analysis (*T* value test), and the comparison between multiple groups used single factor variance (one-way ANOVA followed by Dunnett's test), and the count data uses a chi-square test, which has certain statistical significance.

## 3. Results

### 3.1. Preoperative Treatment

After continuous somatostatin pumping and decompression tube treatment through anorectal obstruction for 4 to 10 days, the average (5.6 ± 1.2) days were compared with the abdominal circumference at admission (100%), and the abdominal circumference before surgery was significantly reduced; it is 81 ± 2.3% (*P* ≤ 0.001). Abdominal CT examination 3 days after comprehensive treatment measured the maximum transverse diameter of the proximal colon to be 2.8 ± 0.3 cm, which was significantly smaller than 6.2 ± 0.5 cm before treatment (*P* ≤ 0.001). In the somatostatin group, after 4 to 7 days and an average of 4.2 ± 1.1 days of treatment, compared with the abdominal circumference at admission (100%), the abdominal circumference before surgery was reduced to 88 ± 1.3% (*P* = 0.01); abdominal CT examination was performed 3 days after treatment to measure the maximum transverse diameter of the proximal colon was 4.6 ± 0.5 cm, which was less than 6.3 ± 0.6 cm before treatment (*P* = 0.02).

### 3.2. Surgical Treatment

All 30 patients underwent surgery. Of these, 13 patients underwent exploratory laparotomy due to unsatisfactory relief of abdominal distension, and the remaining 17 patients underwent laparoscopic exploratory surgery. Of all the patients, 10 patients completed radical surgery with one-stage anastomosis, including 7 patients who underwent laparoscopic surgery. In the remaining 20 cases, the colon was still significantly dilated and edema during operation, and the tumor was excised and the proximal colostomy was performed.

All patients had no complications such as anastomotic leakage, postoperative bleeding, and abdominal infection. All patients in the somatostatin treatment group underwent surgical treatment, and only 5 patients underwent radical tumor resection and one-stage anastomosis during operation. None of the 5 patients underwent anastomosis under laparoscopy, and 1 of 5 patients developed intestinal fistula 6 days after surgery. He was discharged after placing an irrigation tube for continuous irrigation treatment. The bloating relief time of the observation group was 2.3 ± 0.5 d, the abdominal pain relief time was 2.1 ± 0.4 d, and the voluntary exhaust time was 2.2 ± 0.1 d; the control group was 3.5 ± 0.7 d, 3.3 ± 0.7 d, and 3.5 ± 0.6 d. The indicators in the research group were significantly lower than those in the control group, and there was a significant difference between the two groups (*P* < 0.05).

### 3.3. Computed Tomography Image Analysis

In order to more intuitively show the effect of somatostatin on patients with intestinal obstruction, this study selected a medical image before and after surgery for comparison and interpretation.  Figure 1 is a CT image of the patient's intestinal obstruction before surgery, and Figure 2 is a CT image of the maximum diameter of the proximal colon before and after the patient's operation.

### 3.4. Segmentation Result

In this paper, a deep neural network structure is proposed, which is an image segmentation model based on a feature mining network. The innovation lies in three aspects: the first is the feature correction unit, which corrects the feature along the direction that is beneficial to the segmentation result. The second is the macro information mining unit, which uses multiscale convolution kernels to scan small-scale features to obtain more spatial location information. The third is the semantic information mining unit, which uses two branches to dig deeper and more detailed features. Experiments show that all three innovations can improve segmentation performance. The segmentation results are as shown in Figure 3.

### 3.5. Comparative Analysis of the Treatment Results of the Two Groups of Patients

The levels of CRP, IL-6, and TNF-*α* in the observation group were significantly lower than those in the control group. There was a significant difference between the groups (*Р* < 0.05). The statistic chart of changes in inflammatory factors is shown in Figure 5.

After treatment, the symptoms of the two groups of patients were alleviated. The treatment effective rate of the observation group was 93.3%, and the treatment effective rate of the control group was 73.3%; we note that *P* < 0.05. The comparison statistical table is shown in Table 1.

Compared with the control group, the disappearance time of clinical symptoms of the two groups of patients was lower than that of the control group, and the patients recovered faster, with statistical significance (*P* < 0.05). The comparison statistical table is shown in Table 2.

The complication rates of the two groups of patients were compared, the incidence of complications in the observation group was significantly lower than the control group, the effect was better, and the difference was statistically significant (*P* < 0.05). The comparison statistical table is shown in Table 3.

## 4. Discussion

Early inflammatory bowel obstruction puncture occurs late in abdominal surgery and is a mechanical intestinal obstruction [21]. The cause of early postoperative inflammatory bowel obstruction is usually caused by prolonged exposure of the intestinal canal or inflammation in the abdominal cavity during the patient's abdominal surgery. The pathogenic mechanism is relatively complex, and most of them are multifactors acting at the same time. Common factors include inflammation, sympathetic nerve inhibition, release of neurotransmitters, hormones, and the use of narcotic drugs, analgesic drugs, etc. [22–24]. Inflammation can cause intestinal edema and hyperemia in patients, leading to intestinal adhesions and formation of intestinal obstruction. There are still no effective preventive measures at present, and the risk is high after surgery. The principle of treatment is generally fasting, correction of water and electrolyte disturbances, and acid-base balance disorders. Drug treatment is generally given adrenal corticosteroids to promote edema resolution, and antisense treatment with antibiotics is also required [25, 26].

Malignant intestinal obstruction caused by distal colon cancer accounts for 88% to 97% of the lower colorectal obstruction [27], and 7% to 28% of colon cancer patients have intestinal obstruction as the first symptom. In recent years, the incidence of colon cancer has increased year by year [28], and the number of patients with acute intestinal obstruction has increased year by year. The main cause of intestinal obstruction is the accumulation of digestive juices in the proximal digestive tract. Therefore, the key to nonsurgical treatment of intestinal obstruction is to reduce the secretion of digestive juice and reduce the accumulation of fluid in the digestive tract. Somatostatin not only inhibits the secretion of various hormones but also reduces the secretion of digestive juices.

Combined application of somatostatin therapy on the basis of total parenteral nutrition can reduce digestive juice secretion by more than 90%. The reduction of digestive juice can reduce intestinal wall edema, improve the condition of intestinal mucosal epithelial ischemia and hypoxia, and reduce capillary permeability [29–31]. Somatostatin can also inhibit the proliferation of tumor cells to a certain extent. In the last century, Japanese scholars reported for the first time the use of transanal obstruction decompression catheter for decompression and drainage of the proximal colon. At present, domestic and foreign scholars tend to use metal stents to expand or place trans-anal intestinal obstruction catheters to relieve the obstruction for a limited period of laparoscopic radical surgery. Compared with intestinal metal stents, transanal obstruction catheters are less expensive, and the probability of perforation and postoperative pain is also lower. It does not cause strong compression of the tumor, so the possibility of tumor spread is reduced.

In this study, after two groups of patients underwent gastric tube decompression, the fluid accumulation in the proximal digestive tract decreased. Combined use of somatostatin therapy can further reduce the secretion of digestive juice and relieve the pressure of obstructive bowel segment. All patients were able to obtain symptom relief before surgery, and the abdominal circumference was significantly reduced, and the degree of intestinal dilatation was also significantly reduced. Elderly patients with long-term intestinal obstruction mostly have intestinal wall congestion and edema and poor blood flow and more often have complications such as anemia, hypoproteinemia, and electrolyte disturbance important. Transanal obstruction catheter can effectively reduce the accumulation of fluid in the proximal large intestine, reduce the edema and expansion of the intestinal canal, and also be used to repeatedly clean the enema to achieve the purpose of preoperative preparation to clean the intestine. Research has shown that the success rate of intestinal obstruction catheter for colorectal cancer complicated with first-stage anastomosis is 84% to 98%, and postoperative incision infection rate and hospitalization time are significantly better than traditional emergency surgery. In this study, the first-stage anastomosis rate and laparoscopic completion rate after treatment with somatostatin and anorectal obstruction catheter were significantly higher than those with somatostatin treatment alone, and there were no serious complications after surgery.

In summary, the use of somatostatin in the treatment of early inflammatory bowel obstruction after acute abdomen surgery can effectively improve the treatment efficiency of patients, reduce the disappearance time of clinical symptoms, have a lower complication rate, and have a significant therapeutic effect, which is worthy of clinical application.

## 5. Conclusion

With the continuous development of modern medical imaging technology, the information contained in the images is becoming more and more abundant. At the same time, the increasing number of tumor patients has also increased the workload of doctors in diagnosis. It takes a lot of time to read an image of a patient, and it is very important to accurately obtain the tumor information in the image to make a clinical diagnosis of the patient. However, because the results produced in the process of manual tumor segmentation will produce different results due to the doctor's experience and medical background and even the final diagnosis results will be inconsistent, the emergence of auxiliary diagnosis can use the high-performance computing server and depth. Learning technology helps doctors complete tumor segmentation and accelerates the doctor's diagnosis process. This paper mainly introduces the basic concepts and principles of tumor segmentation, traditional segmentation methods, and segmentation methods based on deep learning. This thesis focuses on improving the accuracy of tumor segmentation (especially for smaller tumors) and the interpretability of tumor segmentation in tumor segmentation and improving the quality of medical aided diagnosis.

In conclusion, somatostatin combined with transanal obstruction catheter is safe and effective for the treatment of elderly patients with malignant intestinal obstruction in the distal colon. After a period of treatment, the patient's symptoms can be effectively relieved, and the conditions for surgical treatment can be created. Subsequent surgical treatment has a higher completion rate of laparoscopic surgery and a first-stage anastomosis power, which reduces the incidence of postoperative complications and alleviates patient's hospital stay and financial burden.

## Figures and Tables

**Figure 1:** CT image of patient's intestinal obstruction: front view (a); side view (b). The images depict the location of the patient's intestinal obstruction.

**Figure 2:** CT image of the largest diameter of the proximal colon: before surgery (a); 3 days after surgery (b); 7 days after surgery (c). Note that the arrow indicates the location of the patient's intestinal obstruction.

**Figure 3:** Visualization of the results of organ segmentation in patients with intestinal obstruction.

**Figure 4:** U-Net network model structure diagram.

**Figure 5:** Statistics of changes in inflammatory factors.

**Table 1:** Comparison of the treatment efficiency of the two groups of patients.

Group (*n*)	Cure	Effective	Invalid	Total efficiency (%)
Observation group (15)	9	5	1	93.3%
Control group (15)	7	4	4	73.3%
*χ* ^2^				4.8118
*P*				0.0283

**Table 2:** Comparison of clinical symptoms disappearing time between two groups.

Group (*n*)	Abdominal pain relief time (d)	Exhaust time (d)	Gastrointestinal decompression (md/d)
Observation group (15)	3.16 ± 1.39	2.66 ± 1.45	254.33 ± 236.07
Control group (15)	5.88 ± 1.84	4.78 ± 1.97	605.29 ± 245.78
*τ*	6.46.5	4.7470	5.6407
*P*	0.001	0.001	0.001

**Table 3:** Comparison of the incidence of complications between the two groups.

Group (*n*)	Celiac infection	Ascites	Incidence (%)
Observation group (15)	1	2	20.0%
Control group (15)	2	4	40.0%
*χ* ^2^			8.5227
*P*			0.0035

## Data Availability

The image data used to support the findings of this study have been deposited in the CVC-Clinic dataset (http://www.cvc.uab.es/CVC-Colon/index.php/databases/).
